The article "Terminal drought and heat stress alter physiological and biochemical attributes in flag leaf of bread wheat" was retracted in 2023. Reasons: compromised peer review; a conflict of interest; concerns about the authorship.

# Terminal drought and heat stress alter physiological and biochemical attributes in flag leaf of bread wheat

**DOI:** 10.1371/journal.pone.0232974

**Published:** 2020-05-13

**Authors:** Abdul Sattar, Ahmad Sher, Muhammad Ijaz, Sami Ul-Allah, Muhammad Shahid Rizwan, Mubshar Hussain, Khawar Jabran, Mumtaz A. Cheema

**Affiliations:** 1 College of Agriculture, Bahauddin Zakariya University, Bahadur Sub-Campus Layyah, Layyah, Pakistan; 2 Cholistan Institute of Desert Studies (CIDS), The Islamia University of Bahawalpur, Bahawalpur, Pakistan; 3 Department of Agronomy, Bahauddin Zakariya University, Multan, Pakistan; 4 Department of Plant Production and Technologies, Faculty of Agricultural Sciences and Technologies, Nigde Omer Halisdemir University, Nigde, Turkey; 5 School of Science and the Environment, Grenfell Campus Memorial University of Newfoundland, Corner Brook, Canada; Harran University, TURKEY

## Abstract

Heat stress along with low water availability at reproductive stage (terminal growth phase of wheat crop) is major contributing factor towards less wheat production in tropics and sub-tropics. Flag leaf plays a pivotal role in assimilate partitioning and stress tolerance of wheat during terminal growth phase. However, limited is known about biochemical response of flag leaf to combined and individual heat and drought stress during terminal growth phase. Therefore, current study investigated combined and individual effect of terminal drought and heat stress on water relations, photosynthetic pigments, osmolytes accumulation and antioxidants defense mechanism in flag leaf of bread wheat. Experimental treatments comprised of control, terminal drought stress alone (50% field capacity during reproductive phase), terminal heat stress alone (wheat grown inside plastic tunnel during reproductive phase) and terminal drought stress + terminal heat stress. Individual and combined imposition of drought and heat stresses significantly (p≤0.05) altered water relations, osmolyte contents, soluble proteins and sugars along with activated antioxidant defensive system in terms of superoxide dismutase (SOD), peroxidase (POD) and ascorbate peroxidase (APX). Turgor potential, POD and APX activities were lowest under individual heat stress; however, these were improved when drought stress was combined with heat stress. It is concluded that combined effect of drought and heat stress was more detrimental than individual stresses. The interactive effect of both stresses was hypo-additive in nature, but for some traits (like turgor potential and APX) effect of one stress neutralized the other. To best of our knowledge, this is the first report on physiological and biochemical response of flag leaf of wheat to combine heat and drought stress. These results will help future studies dealing with improved stress tolerance in wheat. However, detailed studies are needed to fully understand the genetic mechanisms behind these physiological and biochemical changes in flag leaf in response to combined heat and drought stress.

## Introduction

Crop growth and productivity are prominently affected by high heat and less water availability [1]. The rise in annual mean temperature around the globe, modification in precipitation patterns and emerging drought risks in many regions have affected agriculture at global level [2], which has imposed limitations on crop yield potential. According to IPCC [3], decreasing water availability and increasing temperature is expected to worsen in coming decades. There is an immense need to identify tolerant plant species and genotypes to these stresses [4,5]. Crop plants at reproductive stages are more susceptible to combined heat and drought stresses than individual ones [1,6]. Drought and heat stress are interlinked; however, researchers usually focus individual effects of both these stresses on plants. It is predicted that global temperature will rise by 1.5 to 4.5 °C until the end of the current century [3]. Lobel et al. [7] predicted 5.5% decrease in global wheat (*Triticum aestivum* L.) production due to these two stresses through simulation modeling. Similarly, Zampieri et al. [8] reported that heat and drought stress results in more concurrent yield anomalies in wheat leading to concerns about global food security.

Drought and heat stress significantly reduce photosynthetic efficiency, stomatal conductance, leaf area and water-use efficiency of cereals, i.e., wheat and maize (*Zea mays* L.) [4,9,10]. Heat stress increases evapotranspiration leading to drought stress in crop plants [11]; thus, water relations of the plants are severely affected under drought stress. Plants opt different mechanisms to respond individual and combined stresses [12,13,14]. For instance, photosynthesis is reduced due to less available moisture and high heat stress, whereas stomata are closed in response to drought stress [9]. Similarly, biochemical reactions are modified under heat stress [15]. The modifications in physiological and gas exchange traits lead to yield reduction. It is reported that seed priming with osmoprotectants can mitigate adverse effects of drought stress [16,17]. Heat stress adversely affects photosynthetic apparatus and assimilate supply duration [18], which lowers yields. Heat stress is also responsible for oxidative stress damage through production of reactive oxygen species (ROS), particularly in chloroplasts in the absence of detoxification system. Chlorophyll molecules experience over-excitation due to high temperature, leading to ROS generation. The ROS generation is clearly observed during leaf senescence process [19].

Plants are equipped with internal defense system equipped with antioxidant enzymes [superoxide dismutase (SOD), catalase (CAT) and peroxidase (POX)] for ROS scavenging under stressed conditions [19]. The combined drought and heat stress modify plant response in a unique fashion compared to individual stress [14,20,21]. Flag leaf of wheat play an important role in carbohydrates assimilation and antioxidant defense mechanism against abiotic stresses like heat and drought [22,23,24]. Luo et al. [22] observed phosphorylation of 58 proteins in wheat due to drought stress out of which 20 were present in flag leaf. Moreover, they reported active role of these proteins in photosynthesis and carbohydrate metabolism. Zhang et al. [24] reported decrease in photosynthetic rate and antioxidant enzymatic activities of flag leaf in response to heat stress coupled with elevated CO_2_. Rivero et al. [14] observed compensatory effect of heat stress on tomato plants under salt stress due to the production of osmoprotectants in response to heat stress. However, such mechanism is still not well identified in wheat. Moreover, to the best of our knowledge, physiological and biochemical responses of flag leaf to combined heat and drought stress have not been reported in literature.

There is a need to identify the plant response mechanism in response to simultaneously occurring heat and drought stress. As flag leaf is a main contributor to the grain yield of wheat; therefore, the aim of current study was to investigate the response of flag leaf of bread wheat in terms of water relations, photosynthetic pigments, osmolytes accumulation and antioxidants defense mechanism against individual and combined drought and heat stress. It was hypothesized that the above-mentioned relations of flag leaf would be more influenced by combined effect of stresses than their individual impacts.

## Materials and methods

### Plant materials and experimental treatments

A pot experiment was conducted to identify the combined and individual effects of terminal drought and heat stress on wheat. Homogenous seeds of variety Faisalabad-2008 (developed by Ayub Agriculture Research Institute Faisalabad Pakistan) were obtained from Agronomic Research Station Karor Lali Ehsan Layyah (31.21° N 70.97° E), Pakistan. The seed was decontaminated with 0.1% (w/v) sodium dodecyl solution and then thoroughly washed using sterilized deionized water. The decontaminated seeds were placed in a clean Petri dish on sterilized filter paper moisturized with distilled water and allowed to grow under shade at room temperature for 5 days. The same sized seedlings were then transplanted to earthen pots (five seedlings to each pot) containing 12 kg of well crushed and sifted soil. Phosphorus (90 mg kg^-1^ P_2_O_5_) as di-ammonium phosphate, potassium (60 mg kg^-1^ K_2_O) as potassium sulphate and nitrogen (100 mg kg^-1^) as urea were comprehensively mixed with soil as basal fertilizer dose. Same amount of NPK was supplied to wheat at tillering stage to maintain the growth. All pots were kept in open space under environmental normal condition until the application of the stress treatments. Drought and heat stress were imposed at BBCH-60 [25] when first anther became visible. Experimental treatments comprised of control (100% field capacity), terminal drought stress (50% field capacity during reproductive stage), terminal heat stress (wheat grown inside the plastic tunnel during reproductive phase) and terminal drought + terminal heat stress.

### Imposition of drought stress

A field capacity (FC; measured on gravimetric basis [26]) was maintained to impose drought stress during reproductive phase. Three soil samples (200 g each) were taken from the soil used to fill the earthen pots. The soil samples were kept at 105 °C for 24 hours. The average weight of these samples was measured to calculate the humidity level before the seed sowing. Three samples (100 g each) from these oven dried soil samples were taken and saturated with distilled water. By calculating the water used for suturing the paste, field capacity was determined as suggested by Nachabe [26]:

$$FC=\frac{Saturation\;percentage\;of\;soil\;sample}{2}$$ (1)

Moisture content of each pot was calculated every day with the help of moisture meter, and irrigation was applied to level the as per calculation. Drought stress was during BBCH-60.

### Imposition of heat stress

Heat stress was imposed during BBCH-60 growth stage of wheat. A plastic tunnel made of transparent polythene sheet was made above the pots by using bamboo sticks. Tiny holes were made in polythene sheet to minimize the humidity. The pots in control treatment were placed under normal conditions [27]. Temperature and humidity were recorded with digital temperature and humidity probe (Digital Multimeter-50302). During heat stress, the temperature of control and heat-stressed pots was recorded twice a day and averaged [28]. The considerable increase in temperature was observed in heat stressed pots in comparison to pots in control treatment (Fig 1).

**Fig 1:** Mean daily temperature of normal and heat stressed treatment for 20 days starting from BBCH 60 growth stage of wheat.

### Water relations

Fresh leaves (W_f_) (0.5 g) were dipped in water till constant weight and weighed (W_S_) to measure the relative water content (RWC). The saturated leaves were then oven dried (80 °C for 24 h) to obtain dry weight (W_d_). The RWC were calculated as suggested by Barrs and Weatherley [29];

$$RWC=\frac{\left(W_{f}-W_{d}\right)}{\left(W_{s}-W_{d}\right)}\times 100$$ (2)

Pressure bomb (Santa Barbara, CA, USA) was used to measure the water potential (Ψw) of fresh leaves. Leaf sample, already used for RWC, was frozen and thawed. S to squeeze the sap and centrifuged (5000 × g). Osmotic potential (Ψs) was measured using an osmometer (Digital Osmometer, Wescor, Logan, UT, USA). The leaf pressure potential (Ψp) was calculated as the difference between Ψw and Ψs.

### Chlorophyll contents

Following the protocol of Arnon [30], fresh leaves (0.5 g) were extracted with 5 mL acetone (80%) by keeping at 0–4 °C for overnight, and centrifuged (10,000 × g) for 5 minutes. The Supernatant was separated and its absorbance was recorded at wavelength 645 and 663 nm using spectrophotometer (Hitachi-U2001, Tokyo, Japan).

### Osmolytes determination

A sample of 0.5 g fresh leaf was taken and grounded in a 1 mL extraction buffer having a pH of 7.2. Sample was prepared by adding cocktail protease inhibitors (1 μM) in the saline phosphate buffer. Saline buffer comprised of 1.37 mM NaCl, 2 mM KH_2_PO_4_, 2.7 mM KCl and 10 mM Na_2_HPO_4_ dissolved in 1 L of deionized water). pH of the buffer was adjusted with HCl and the sample was autoclaved. The extract obtained from sample was centrifuged (12000 × g) for 5 min to separate the supernatant and was stored for determination of the total of soluble proteins by following Bradford assay [31]. Bovine serum albumin with different dilutions (10, 20, 30, 40, 50, 60, 70, 80, 90 and 100 μg μL^-1^) was used to construct standard curves. After adding 400 μL deionized water and Dye stock, sample tubes were vortexed and incubated at room temperature for 30 minutes followed by recording of the sample absorbance using UV 4000 UV-VIS spectrophotometer. Proline was determined by following the method suggested by Simaei et al. [32]. Fresh leaf samples of 0.5 g were homogenized with 10 mL of sulphosalicylic acid (3% w/v) and filtered. The filtrate was taken in test tubes and treated with ninhidrine (2.5%) and glacial acetic acid and were kept in water bath (100 °C for 60 min) for color development. For chromophores separation, toluene was added to test tubes after removal from water bath and ice bath. Optical density (520 nm) was recorded using ultraviolet visible spectrophotometer. The soluble sugar contents were determined by following the method as described by Giannakoula et al. [33].

### Enzymatic antioxidants activities

The 5 ml phosphate buffer (50 mM with 7.8pH) was used for determining the activities of enzymatic antioxidants from centrifuged fresh and healthy leaf sample (15000 × g for 20 min).

Activity of antioxidant enzyme Superoxide dismutase (SOD) was determined at 560 nm as result of photochemical reduction [34]. The reaction mixture comprised of 50 μL enzyme extract, 1 mL NBT (50 μM), 1 mL riboflavin (1.3 μM), 500 μL EDTA (75 mM), 500 μL methionine (13 mM) and 950 μL phosphate buffer (50 mM). The reaction mixture was withheld under the light of 30 W fluorescent lamp to initiate the reaction which was then stopped after 5 minutes by turning of the lamp. The NBT photo reduction caused blue form azane formation, which was read at 560 nm. The blank reading was taken using same reaction mixture lacking enzyme extract. To initiate the reaction for catalase (CAT) activity, 100 μL enzyme extract was mixed into the reaction mixture [900 μL H_2_O_2_ (5.9 mM) and 2 mL phosphate buffer (50 mM)]. The change in the absorbance of H_2_O_2_ produced as a result of CAT activity was measured with the help of UV-visible spectrophotometer at 240nm and was described as μmol of H_2_O_2_ minute^-1^ mg^-1^ of protein [35]. Kar and Mishra [36] procedure was followed the measure the peroxidase (POD) activity. The reaction mixture for peroxidase (POD) was composed of 5 ml of 10mM pyrogallol, 5 ml of 5m MH_2_O_2_, 100 μl enzyme extract and 5 ml of 0.1M Tris-HCL buffer. The POD activity was determined by recording the decline in the absorbance due to the H_2_O_2_ dependent oxidation of pyrogallol at 425 nm and was expressed POD IU minute^-1^ mg^-1^ of the protein.

### Statistical analysis

Data collected were tested for normality using Shapiro-Wilk normality test, which indicated a normal distribution. Therefore, Fisher’s Analysis of Variance (ANOVA) technique considering the completely randomized design was used to test the significance in data. Least Significant Difference (LSD) test (5% probability level) was applied for means comparison where ANOVA indicated significant differences [37]. All statistical computations were performed on Statistix software version 10. Figures were prepared by using bar chart function of Microsoft Excel v. 365.

## Results

### Water relations

Drought and heat stress notably affected the transport of water and solutes. The percentage of relative water contents (RWC) significantly differed among various treatments (Fig 2A). The highest percentage of RWC was observed in control treatment, whereas combined drought and heat stress notably decreased (42%) RWC compared to control. However, individual drought and heat stress resulted in 23 and 25% reduction in RWC as compared to control. Moreover, there was no significant difference between both individual stresses regarding reduction in RWC (Fig 2A). Water potential (WP) was enhanced (67%) by combined stresses as compared to control. The lowest values of WP were observed for control treatment (Fig 2B). Osmotic potential (OP) increased with stress exposure. The highest osmotic potential value (1.47 -MPa) was observed under combined stresses as compared to control (0.89 –Mpa) (Fig 2C). The individual drought stress resulted in more osmotic potential as compared to individual heat stress and control (Fig 2C). The highest turgor potential (TP) was observed in control treatment (0.52 MPa), while the lowest was noted under heat stress (0.23 MPa). Moreover, drought stress decreased TP (by 34%), and combined stresses reduced TP (by 36.5%) as compared to control (Fig 2D).

**Fig 2:** Effects of different drought and heat treatments on relative water content (A), Water potential (B), Osmotic potential (C) and Turgor Potential (D) of wheat. Values shows mean ± SE (n = 3). Bars sharing the same letters are statistically at par with each other at significance level of 5% (*P*≤0.05).

### Photosynthetic pigments

The chlorophyll was significantly influenced by imposed stresses (Fig 3). The reduction in chlorophyll a content was 51.6%, 55.5% and 55% under drought, heat and combined stresses, respectively compared to control treatment (Fig 3A). However, combined stresses resulted in the highest reduction of chlorophyll b contents (67%) as compared to control. Drought and heat stress resulted 56 and 47.8% reduction in decreased chlorophyll content as compared to control (Fig 3B). The highest (3.40 mg g^-1^ FW) and the lowest (1.42 mg g^-1^ FW) Chlorophyll a+b was values were recorded for control and combined stress treatments, respectively (Fig 3C). The chlorophyll a/b content was significantly increased with combined stresses (27%), as compared to control (Fig 3D).

**Fig 3:** Effects of different drought and heat treatments on chlorophyll a (A), chlorophyll b (B), chlorophyll a+b (C) and chlorophyll a/b (D) of wheat. Values show mean ± SE (n = 3). Bars sharing the same letters are statistically at par with each other at significance level of 5% (*P*≤0.05).

### Osmolytes

The proline contents were increased with imposed stresses with the highest increase (69.8%) under combined stresses compared with control. Individual drought and heat stress resulted in 53% and 58.9% increase in proline contents as compared to control (Fig 4A). Soluble protein was also influenced by imposed stresses with minimum values observed under control treatment (Fig 4B).

**Fig 4:** Effects of different drought and heat treatments on proline (A), soluble protein (B) and soluble sugar (C) of wheat. Values show mean ± SE (n = 3). Bars sharing the same letters are statistically at par with each other at significance level of 5% (*P*≤0.05).

An increase of 3.6 mg g^-1^, 4.3 mg g^-1^ and 4.5 mg g^-1^ in soluble protein was recorded under drought, heat and combined stresses, respectively as compared to control treatment. The minimum value of soluble sugar (1.46 mg g^-1^) was observed for control treatment, while combined stresses resulted in 4.55 mg g^-1^ soluble sugar. The individual drought and heat stresses resulted in 61 and 62% increase in soluble protein as compared to control (Fig 4C).

### Enzymatic antioxidants activities

The imposed stresses induced the catalase activity as compared to control treatment. The highest catalase activity (61%) was measured under combined stresses (Fig 5A).

**Fig 5:** Effects of different drought and heat treatments on Catalase (A), Superoxide dismutase (B), Peroxidase (C) and Ascorbate peroxidase (D) of wheat. Values show mean ± SE (n = 3). Bars sharing the same letters are statistically at par with each other at significance level of 5% (*P*≤0.05).

The superoxide dismutase (SOD) activity was significantly increased with exposure of stresses and the highest SOD activity (54%) was observed under combined stresses. The lowest SOD activity was noted in control treatment (Fig 5B). The highest peroxidase (POD) activity was determined under individual drought stress, followed by combined stresses (Fig 5C).

The ascorbate peroxidase activity was induced with imposed stresses as compare to control. The maximum increase (68%) in ascorbate peroxidase was observed under drought stress. Heat stress and combined stresses resulted in 39 and 55% increase in ascorbate peroxidase activity as compared to control.

## Discussion

Relative water content is considered as an indication of water condition of cell and correlated with biotic and abiotic stresses, including drought and heat stress. Relative water content and water potential are regarded as the better indicator of drought stress as compared to other biochemical and physiologically features of plants [9,38]. Results indicated that drought and heat stress (either alone or combined) were found detrimental to water related parameters. Moreover, when plants were exposed to combined drought and heat stress, they showed lower relative water relations as compared to individual stresses. Negative impact of drought and heat stress on water relations of the plants has been reported by many researchers [9,38]. The decrease in relative water relations was due to enhanced transpiration in stressed leaf and reduced osmotic potential [38, 39]. The more detrimental effects on plant relative water relations were observed due to combined drought and heat stresses as compared to their individual effects. The higher reduction in relative water relation under combined stresses can be attributed to lower water use efficiency of plant under water deficit conditions. Drought stress significantly reduced water use efficiency of wheat as compared to well-watered conditions [10,16]. Heat stress damaged plants root conductance despite enough supply of water, while this becomes more fatal for plant when heat stress along with drought was applied due to more water transpiration demands.

Combined stresses exerted negative effects on all water relation parameters except turgor potential (Fig 2D). Improvement in turgor potential with combined stresses contrasted with expected results. The accumulation of secondary metabolite and osmolytes produced in response to heat stress probably reduced turgor potential [14, 39]. However, a reduction in other water relations i.e. osmotic potential, RWC, turgor pressure, was found with combine stresses, which still needs to be explored.

The significant decrease in pigment contents was due to exposure of drought and heat stresses, while reduction was increased under combined stresses. The photo-inhibition and photo-destruction of pigments and related protein complexes, and disruption of photosynthetic membrane both are caused by drought stress [39,40]. Decreased chlorophyll content under drought stress is usually attributed to the destruction of various enzymes involved in the synthesis of chlorophyll and enhanced activity of enzymes that degrade the chlorophyll content [39,41], while heat stress causes reduction in chlorophyll content by destroying thylakoid membranes [42, 43]. Therefore, minimum build-up of chlorophyll contents in plants might be due to increased degradation or decreased biosynthesis of chlorophyll contents or integrated effect of both under heat stress. Moreover, water deficit condition may alter plant physiological and biochemical processes (photosynthesis, respiration, ion uptake, translocation, nutrient metabolism, carbohydrate assimilation, and growth promoters), resultantly damaged plant growth [9,18,26].

Plants affected by drought and heat stress had confirmed the accretion of compatible solute such soluble sugars and proline [14,38,39]. In the present study, enhanced proline content were observed under combined stresses as compared to individual stresses. The increased accumulation of proline due to drought and heat stress has been reported by the researchers who concluded that proline helps to stabilize membranes, sub-cellular structures and cellular redox potential by destroying the free radicals [39,38,44,45]. Increase in soluble protein content was also observed under combined stresses; however, the production was more pronounced under heat stress [46,47]. Increase in soluble protein contents might be attributed to the enhanced production of amino acids that were produced in response to heat or drought stress. Jin et al. [48] reported the accumulation of certain amino acids (glutamine, ornithine, valine tryptophan and tyrosine,) in purslane plants in response to combined drought and heat stress. Significant increase in soluble sugar contents was observed in plants subjected to drought and heat stress (both alone and combine) as compared to control (no stress). However, impact of drought and heat stress was non-significant when compared to each other. Soluble sugars contents and sucrose synthase activity were increased with stress exposure; hence, soluble sucrose content was also increased [46,47,49,50]. Liu et al. [49] observed a significant increase in starch content under heat shock treatment above 30 °C. Increased sucrose content might be due to the activation of enzymes that resulted in the breakdown and remobilization of starch [51,52] to release energy and to help mitigate the effect of stress.

Response of enzymatic activities varied with different stresses, i.e., alone or combined. Drought or heat stress enhances the activities of antioxidants despite these were applied as alone or in combination. The activities of catalase, peroxidase, superoxide dismutase and ascorbate peroxidase were increased with exposure to drought and heat stress either alone or combine [14,52,53]. The generation of destructive reactive oxygen species, including superoxide radical (O^2−^), singlet oxygen (^1^O_2_), hydroxyl radical (OH^−^) and hydrogen peroxide (H_2_O_2_)was probably the reason of enhanced enzyme activities [13,14,54,55]. Production of ROS often induce the production of abscisic acid that is signal molecule under stressed conditions and regulate the gene expressions that control the production of enzymatic antioxidants such as superoxide dismutase and catalase [9,52]. Peroxidase and ascorbate peroxidase activities were reduced when drought stress was combined with heat stress as compared to sole drought stress. This improvement may be attributed to accumulation of secondary metabolite and osmolytes produced in response to heat stress [14,38,39], which resulted in reduction of peroxidase and ascorbate peroxidase activities as compared to drought stress alone. The reduction in other enzymatic activities under combined stresses needs to be explored.

## Conclusion

Wheat has potential to maintain its growth and development under individual or combined drought and heat stress by altering physiological and biochemical attributes. Turgor potential was lowest under heat stress, while comparative improvement was observed when drought stress was combined with heat stress. Similarly, heat stress exerted compensatory effect on peroxidase and ascorbate peroxidase activities of flag leaf under drought stress. Moreover, combined stresses resulted in disturbed water relation and chlorophyll content and increased osmotic potential, proline, soluble protein and soluble sugar contents, catalase and superoxide dismutase activities as compared to individual stress. The interactive effect of both stresses was hypo-additive in nature, but for some traits (like turgor potential and APX) effect of one stress neutralized the other. These results will help future studies dealing with improved stress tolerance in wheat. However, detailed studies are needed to fully understand the genetic mechanisms behind these physiological and biochemical changes in flag leaf in response to combined heat and drought stress.
